# Effect of Chronic Exposure to Prometryne on Oxidative Stress and Antioxidant Response in Red Swamp Crayfish (*Procambarus clarkii*)

**DOI:** 10.1155/2014/680131

**Published:** 2014-03-18

**Authors:** Alžběta Stará, Antonín Kouba, Josef Velíšek

**Affiliations:** University of South Bohemia in Ceske Budejovice, Faculty of Fisheries and Protection of Waters, South Bohemian Research Center of Aquaculture and Biodiversity of Hydrocenoses, Research Institute of Fish Culture and Hydrobiology, Zatisi 728/II, 389 25 Vodnany, Czech Republic

## Abstract

The aim of the study was to investigate effects of the triazine herbicide prometryne on red swamp crayfish on the basis of oxidative stress, antioxidant indices in hepatopancreas and muscle, and histopathology of hepatopancreas. Crayfish were exposed to prometryne concentrations of 0.51 **μ**g L^−1^, 0.144 mg L^−1^, and 1.144 mg L^−1^ for 11 and 25 days. Indices of oxidative stress (thiobarbituric acid reactive substances (TBARS)), and antioxidant parameters (superoxide dismutase (SOD), catalase (CAT), and glutathione reductase (GR)) in crayfish muscle and hepatopancreas were measured. Chronic exposure to prometryne did not showed the impact of oxidative damage to cells. Changes activity of the antioxidant enzymes SOD, CAT, and GR were observed in all tested concentrations to prometryne for 11 and 25 days (*P* < 0.01) as compared with the control group. We did not see any differences in histopatological examination to hepatopancreas. Prolonged exposure of prometryne did not result in oxidative damage to cell lipids and proteins, but it led to changes in antioxidant activity in crayfish tissues. Changes in antioxidant systems were also observed in the environmental prometryne concentration of 0.51 **μ**g L^−1^. The results suggest that antioxidant responses may have potential as biomarkers for monitoring residual triazine herbicides in aquatic environments.

## 1. Introduction

The increasing worldwide contamination of surface and groundwater systems with thousands of industrial and natural chemical compounds is one of the key environmental problems today [1]. Pesticides are one of the main components contributing to the pollution of aquatic ecosystems. Pesticides are used to control the live organisms in agriculture. However, there is compelling evidence that agricultural pesticide use has a major impact on water quality as it can cause extensive pollution of drinking water, such as rivers, lakes, and estuaries, and together they are affecting also nontarget aquatic organisms [2–4].

Prometryne, 2,4-bis(isopropylamino)-6-methylthio-s-triazine, a selective herbicide of the s-triazine family, has been used as a pre- or postemergence controller of annual grasses and broadleaf weeds in a variety of crops [5, 6]. Prometryne is an inhibitor of photosynthesis by inhibiting electron transport in targeted broad-leaved plants and grasses [7]. Because of its poor absorption in the soil, it is easily breaking down through this matrix and contaminates the groundwater [8].

Although prometryne has been banned in Europe since 2004 [9], it still can be found in surface and ground waters. Prometryne was reported in groundwater of Greece at concentration exceeding 1 *μ*g L^−1^ [10] and in surface water it has been reported at concentrations from 0.190 to 4.40 *μ*g L^−1^ [11]. In surface water of Western France, remains of prometryne were detected at concentrations from 0.1 to 0.44 *μ*g L^−1^ [12]. In case of the Czech rivers, the maximum environmental concentration of prometryne 0.51 *μ*g L^−1^ was detected [13]. But nevertheless prometryne is still being widely used in China [9], Australia, Canada, New Zealand, South Africa, and the United States [14].

Prometryne poses an acute risk to nontarget aquatic organisms. Based on acute toxicity tests, it is slightly to moderately toxic to aquatic plants, zooplankton, and fish. Five-day EC50 of prometryne is 0.023 mg L^−1^ for algae* Selenastrum capricornutum* [5], 24hEC50 is 0.083 *μ*mol L^−1^for common duckweed (*Lemna minor*)^,^ and 24hLC50 is 0.071 *μ*mol L^−1^ for bearded stonewort (*Chara canescens*) [15]. For water flea (*Daphnia pulex*), the average toxicity to prometryne is 96hLC50 40 *μ*g L^−1^ [5]. Acute toxicity (96hLC50) in rainbow trout (*Oncorhynchus mykiss*) is 2.9 mg L^−1^ [16] and for common carp (*Cyprinus carpio*) is 8 mg L^−1^ [17]. Effect of chronic toxicity to prometryne on nontarget aquatic organisms has not been investigated to a significant extent. Some studies are dealing with fish, for example, fathead minnows (*Pimephales promelas*) [7] and various early live stages of common carp [18–20].

The main objective of this study was to evaluate the effects of chronic toxicity to prometryne on nontarget organisms. In this study, red swamp crayfish (*Procambarus clarkii*) was selected. Crayfish are an ecologically important benthic invertebrates in the environment, and they are considered an appropriate model organisms [21, 22]. The main aim was observing antioxidant activity changes and oxidative damage in the hepatopancreas and abdominal muscle of crayfish after long-term exposure to differing prometryne concentrations. Oxidative stress and antioxidant systems are considered as good indicators of xenobiotic accumulation in fish tissue [18, 19], and on crayfish these studies were not yet performed. Also, we observed the behavior of crayfish and examinated hepatopancreas histopathologically. Furthermore, the effects of acute, subchronic, and chronic exposure of fish to triazine herbicides have been documented. But on the other hand, there is a scarcity of data on the chronic exposure to these compounds at real environmental concentrations with respect to oxidative stress and antioxidant responses in the macroinvertebrates.

## 2. Materials and Methods

### 2.1. Chemical

High-purity-certified standard of prometryne (2,4-bis(isopropylamino)-6-methylthio-s-triazine) (99.3%) was purchased from Sigma Aldrich, Czech Republic.

### 2.2. Experimental Animals

European native species of crayfish are endangered and thus they should be protected. For our study, we have chosen the invasive species red swamp crayfish (*Procambarus clarkii*) as a model species. Crayfish (mean carapace length 28.53 ± 1.61 mm, postorbital carapace length 23.61 ± 2.31 mm, and weight 5.9 ± 1.08 g) were held in aquaria containing 100 L of freshwater with continuous aeration, at 19–23°C and a 12L:12D cycle. Dissolved oxygen concentration measured daily was 90–98%, and pH was 7.5 ± 0.3. Aquariums were equipped with plastic shelters to deter cannibalism [23]. Crayfish were acclimatized for 10 days before the beginning of the experiment.

### 2.3. Experimental Protocol

The experiment was a semistatic method conducted over 25 days. Red swamp crayfish were allocated, in groups of 12, to one of three experimental regimes or to an untreated control group. The experimental fish were exposed to prometryne at the following concentrations: 0.51 *μ*g L^−1^ (the reported environmental concentration in Czech rivers [13]), 0.144 mg L^-1,^ and 1.144 mg L^−1^. Concentrations of 0.144 mg L^−1^ and 1.144 mg L^−1^ corresponded to 1% of the 96hLC50 and 10% of 96hLC50 for signal crayfish (*Pacifastacus leniusculus*) (the only one crayfish species examined in acute toxicity test on prometryne [24]). The experimental conditions were duplicated for a total of eight groups (*n* = 96). Crayfish were fed experimental diet containing fish meal 40%, wheat flour 38%, soybean flour 10%, cornstarch 10%, vitamin and mineral premix 1%, fish oil 0.5%, and rapeseed oil 0.5% at 1% body weight per day in two feeding doses. Eighty percent of the exposed solution was renewed each day 2 h after feeding to maintain water quality and the appropriate concentration of prometryne.

During the experiment, crayfish behavior and survival rate were recorded. To ensure agreement between nominal and actual compound concentrations in the aquaria, water samples were analyzed during the experimental period by LC-MS/MS [25]. Water samples were collected from the aquaria 1 h and 24 h after renewing the test solutions. The mean concentration of prometryne in the water samples was always within 5% of the intended concentration.

### 2.4. Tissue Samples and Preparation of Postmitochondrial Supernatant

At the completion of each exposure period (11 and 25 days), three crayfish from each aquarium were randomly selected and killed. The hepatopancreas and abdominal muscle were quickly removed, immediately frozen, and stored at −80°C for analysis. Frozen tissue samples were weighed and homogenized (1 : 10, w/v) with an Ultra Turrax homogenizer (Ika, Germany) using 50 mM potassium phosphate buffer, pH 7.0, containing 0.5 mM EDTA. The homogenate was divided into two portions, one to measure thiobarbituric acid reactive substances (TBARS) and the other, centrifuged at 12 000 g for 30 min at 4°C, to obtain the postmitochondrial supernatant for other antioxidant parameter analyses.

### 2.5. Indices of Oxidative Stress and Antioxidant Parameters

The TBARS method described by Lushchak et al. [26] was used to evaluate lipid peroxidation. The superoxide dismutase (SOD; EC 1.15.1.1) activity was determined by the method of S. Marklund and G. Marklund [27]. This assay depends on the autoxidation of pyrogallol. Superoxide dismutase activity was assessed spectrophotometrically with a spectrophotometer Tecan (Infinite M200 Tecan, Switzerland) at 420 nm and expressed as the amount nmoles NBT per milligram of protein. The catalase (CAT; EC 1.11.1.6) activity assay, using the spectrophotometric measurement of H_2_O_2_ breakdown at 240 nm, was performed following the method of Beers and Sizer [28]. Glutathione reductase (GR) activity was determined spectrophotometrically, measuring NADPH oxidation at 340 nm [29].

### 2.6. Protein Content Determination

Total protein content in each sample was determined spectrophotometrically according to the method of Bradford [30] using bovine serum albumin as a standard.

### 2.7. Histopathology

Histopathological examination of crayfish hepatopancreas was performed at the end of toxicity test, after 25 days. The taken samples of hepatopancreas were immediately fixed in 10% formalin, drained, and embedded in paraffin. Sections were made of the paraffin blocks, stained with hematoxylin-eosin, examined by light microscopy, and photographed using a digital camera.

### 2.8. Statistical Analysis

The statistical software program STATISTICA (version 8.0 for Windows, StatSoft) was used to compare differences among the test groups. Prior to analysis, all measured variables were checked for normality (Kolmogorov-Smirnov test) and homoscedasticity of variance (Bartlett's test). If these conditions were satisfied, a one-way analysis of variance (ANOVA) was employed to determine differences in measured variables among experimental groups. When a significant difference was detected (*P* < 0.01), Dunnett's multiple range test was applied. If the conditions for ANOVA were not satisfied, a nonparametric test (Kruskal-Wallis) was used [31].

## 3. Results and Discussion

Laboratory studies of oxidative stress, antioxidant enzymes, and histopathological responses in tissues of crayfish exposed to herbicides can provide information on and help to elucidate the mechanisms of the impact of residual herbicides on crayfish. The results of this study provide further data on long-term exposure to prometryne for consideration in risk assessment. The findings contribute to knowledge of the toxic potential of prometryne to red swamp crayfish at actual concentrations in Czech rivers.

### 3.1. Crayfish Behavior during the Experiment

During the experiment, both control and exposed to prometryne crayfish showed normal feeding behavior. There were no signs of respiratory distress, increased rate of movement activities, or floating. To our knowledge, no other data on behavior of crayfish after triazine exposure are available in the literature. Buric et al. [22] reported excited behavior (fast and chaotic movement outside the shelters, specimens attempting to “escape”) in crayfish following acute poisoning with diazinon (0.3–0.5 *μ*g L^−1^). In the acute course of triazines poisoning in fish, the following clinical symptoms are typical: accelerated respiration, loss of movement coordination, and alternating the resting phase to the excitation phase, and at the end, they fall into damp and move mainly on their flanks, their respiration slowed down, and the damp phase and subsequent agony are very long [32]. In chronic toxicity tests, any changes in fish behavior have not been shown [33], and also in the test on prometryne [18, 19], like in our tests on crayfish.

### 3.2. Indices of Oxidative Stress and Antioxidant Parameters

The damage of tissues and cellular components is the result of oxidative stress, due to the oxygen-free radicals and other reactive oxygen species [34]. The use of antioxidant defense enzyme activities before oxidative damage in aquatic organisms as molecular biomarkers of environmental pollution has been proved to be of great diagnostic value [35]. The effect of chronic exposure to prometryne on TBARS level in red swamp crayfish tissues is shown in Table 1. In this study, any significant differences in lipid peroxidation level among exposed groups were not observed.

Oxidative substances in cells may lead to an elevation of antioxidant enzymes as a defense mechanism. Induction of antioxidant enzymes is an important line of defense against oxidative stress in biological systems [36]. The organisms have their own cellular antioxidative defense system, composed of both enzymatic and nonenzymatic components [37]. Antioxidant defense system is mainly constituted of superoxide dismutase, catalase, and glutathione dependent enzymes (glutathione peroxidase, glutathione reductase, and glutathione-S-transferase) [38]. The SOD is a group of metalloenzymes that play a crucial role as antioxidants and constitute the primary defense system against the toxic effects of superoxide radicals (O_2_^−^) in organisms [39, 40]. Significant differences from the control value (*P* < 0.01) in the SOD activities were seen at all exposure durations to prometryne in hepatopancreas after exposure of 11 days (Table 2). In hepatopancreas, we observed significantly decreased SOD activities in concentrations to prometryne 0.144 and 1.44 mg L^−1^ compared to control group at the end of the test. The SOD activity was observed significantly to be lower in muscle in concentration of prometryne 0.144 and 1.44 mg L^−1^ compared with control group after 25 days. The CAT is an enzyme which facilitates the removal of hydrogen peroxide (H_2_O_2_), onto molecular oxygen and water [41]. The CAT activity in our test was significantly (*P* < 0.01) decreased in the groups tested, 0.144 and 1.44 mg L^−1^ prometryne at 11 days, and in all tested groups after 25 days of exposure (Table 3). Glutathione reductase (GR) plays an essential role in cell defense against reactive oxygen metabolites. GR maintains the reduced status of glutathione, whose reducing power is also necessary for gluthatione peroxidase activity and so GR keeps of overall homeostatic oxido-reductive balance in any living cell [42]. The GR activity was observed significantly (*P* < 0.01) to be lower in hepatopancreas and higher in muscle after 25 days of all exposed groups compared to the control group (Table 4).

These oxidative stress and antioxidant enzymes changes have not yet been well documented in crayfish, but there are a number of studies on the effect of triazine herbicides on fish. Stara et al. [19] investigated changes in antioxidant systems against oxidative damage of tissues (muscle, brain, intestine, liver, and gills) in common carp after 60-day exposure to prometryne, also in the environmental concentration of 0.51 *μ*g L^−1^. Jin et al. [43] examine the effects of atrazine on zebra fish (*Danio rerio*) for 14 days. Fish have increased SOD activity (at the concentrations of 0.1 and 1 mg L^−1^ atrazine) and CAT (in the concentration of 1 mg L^−1^ of atrazine) in the liver. A similar result was demonstrated in an experiment to terbutryn in tissues common carp after 90 days. Velisek et al. [44] observed significant higher SOD activities in brain and liver, and the GR activity was lower in liver and intestine, and higher in muscle.

In summary, in this study, it has been found that the antioxidant enzymes (SOD, CAT, and GR) maintain a balance in cells and protect them from oxidative damage tissues (hepatopancreas, muscle) of crayfish after chronic exposure of the triazine herbicide prometryne after 11 and 25 days, it also in environmental concentration 0.51 *μ*g L^−1^. Thus, we could suggest that some antioxidants changes in crayfish tissues, which were contaminated by prometryne, could occur as an adaptive mechanism to this stressful situation. At the same time, we must not forget that the antioxidant defense is involved a number of other enzymes, and oxidative stress may influence other factors such as species, habitat, and the feeding behavior.

### 3.3. Histopathological Examination

No histopathological changes were demonstrated in hepatopancreas of red swamp crayfish following chronic exposure to prometryne at all tested concentrations. For the crayfish, the effect of chronic exposure to pesticides at low concentrations on histopathological changes in tissues has not yet been studied (monitored). Some studies describe histopathological changes in crayfish tissues after acute exposure to some pesticides. For example, Desouky et al. [45] reported extensive ultrastructural alterations to hepatopancreas epithelial cells, the most notable pathological features including vacuolation, degradation, and distinct cell lysis in red swamp crayfish following acute exposure with insecticide ethion (0.36 mg L^−1^). However, the long-term effect of triazine herbicides is well documented on fish. Study on the common carp was most prominent in prometryne concentrations of 8 and 80 *μ*g L^−1^ after 60 days of treatment, when were observed histopathological changes severe hyaline degeneration of the epithelial cells of caudal kidney tubules in fish [24].

## 4. Conclusion

To our knowledge, this is the first report of the effects of triazine herbicide study, respectively prometryne with using oxidative parameter and antioxidants biomarkers on the crayfish. Crayfish was used as one with sensitive nontarget aquatic organisms exposed to various pollutants in the environment. Moreover, during the study behavior of crayfish was monitored and the histopathological examination was performed in the hepatopancreas at the end of the test. The information presented in this study will be helpful in fully understanding the mechanism of effect of prometryne on the crayfish.

## Figures and Tables

**Table 1:** Effect of chronic exposure to prometryne on level of thiobarbituric acid reactive substances (TBARS, nmol mg^−1^ protein) in red swamp crayfish tissues.

Indices	Exposure time (days)	Test groups			
		Control	Prometryne 0.51 *μ*g L^−1^	Prometryne 144 mg L^−1^	Prometryne 1.44 mg L^−1^
Hepatopancreas	11	0.535 ± 0.04	0.515 ± 0.03	0.614 ± 0.09	0.614 ± 0.07
	25	0.521 ± 0.09	0.538 ± 0.06	0.479 ± 0.04	0.495 ± 0.06

Muscle	11	0.594 ± 0.08	0.576 ± 0.10	0.619 ± 0.12	0.712 ± 0.19
	25	0.669 ± 0.11	0.650 ± 0.13	0.704 ± 0.06	0.681 ± 0.06

Data are means ± SD, *n* = 6.

**Table 2:** Effect of chronic exposure to prometryne on superoxide dismutase (SOD, nmol NBT min^−1^ mg^−1^ protein) activity in red swamp crayfish tissues.

Indices	Exposure time (days)	Test groups			
		Control	Prometryne 0.51 *μ*g L^−1^	Prometryne 0.144 mg L^−1^	Prometryne 1.44 mg L^−1^
Hepatopancreas	11	0.216 ± 0.01	0.111 ± 0.05*	0.126 ± 0.02*	0.132 ± 0.04*
	25	0.164 ± 0.04	0.155 ± 0.04	0.086 ± 0.02*	0.076 ± 0.02*

Muscle	11	0.075 ± 0.04	0.057 ± 0.03	0.093 ± 0.06	0.098 ± 0.17
	25	0.330 ± 0.01	0.043 ± 0.02	0.008 ± 0.00*	0.010 ± 0.00*

Data are means ± SD, *n* = 6. Significant differences compared with control value, *<0.01.

**Table 3:** Effect of chronic exposure to prometryne on catalase (CAT, *μ*mol H_2_O_2_ min^−1^ mg^−1^ protein) activity in red swamp crayfish tissues.

Indices	Exposure time (days)	Test groups			
		Control	Prometryne 0.51 *μ*g L^−1^	Prometryne 0.144 mg L^−1^	Prometryne 1.44 mg L^−1^
Hepatopancreas	11	4.018 ± 0.78	4.098 ± 0.59	1.695 ± 1.10*	1.065 ± 0.84*
	25	3.953 ± 1.06	2.073 ± 0.69*	1.515 ± 0.60*	0.834 ± 0.40*

Muscle	11	0.121 ± 0.06	0.105 ± 0.04	0.106 ± 0.04	0.112 ± 0.07
	25	0.150 ± 0.03	0.149 ± 0.02	0.116 ± 0.05	0.146 ± 0.04

Data are means ± SD, *n* = 6. Significant differences compared with control value, *<0.01.

**Table 4:** Effect of chronic exposure to prometryne on glutathione reductase (GR, nmol NADPH min^−1^ mg^−1^ protein) activity in red swamp crayfish tissues.

Indices	Exposure time (days)	Test groups			
		Control	Prometryne 0.51 *μ*g L^−1^	Prometryne 0.144 mg L^−1^	Prometryne 1.44 mg L^−1^
Hepatopancreas	11	1.250 ± 1.47	0.300 ± 0.19	0.272 ± 0.17	0.249 ± 0.11
	25	1.221 ± 0.58	0.489 ± 0.31*	0.418 ± 0.11*	0.314 ± 0.17*

Muscle	11	0.308 ± 0.23	0.337 ± 0.11	0.745 ± 0.42	0.623 ± 0.13
	25	0.307 ± 0.18	0.608 ± 0.19*	0.646 ± 0.16*	0.660 ± 0.07*

Data are means ± SD, *n* = 6. Significant differences compared with control value, *<0.01.
